# Research on Urban National Sports Fitness Demand Prediction Method Based on Ant Colony Algorithm

**DOI:** 10.1155/2022/5872643

**Published:** 2022-04-07

**Authors:** Wei Yue, Peng Dai

**Affiliations:** ^1^College Physical Education Department, Qingdao Huanghai University, Qingdao, Shandong 266427, China; ^2^Dean's Office, Qingdao Binhai University, Qingdao, Shandong 266427, China

## Abstract

With the development of competitive sports, the enthusiasm of the public to participate in sports has gradually increased. At present, almost all streets in the city have their own fitness places, which provide a lot of help for public fitness. However, the existing fitness venues are obviously insufficient, the venues are limited, relatively single, and the open-space area is insufficient, which cannot meet the needs of mass sports fitness. Based on this, this paper studies and analyzes the prediction of urban national sports fitness demand based on the ant colony algorithm. First, this paper analyzes the National Fitness Situation and the related research on demand forecasting and puts forward the use of the ant colony algorithm to realize demand forecasting. This paper expounds on the research methods and algorithms commonly used in demand forecasting. The ant colony algorithm is used to improve the fuzzy analysis. The urban national sports fitness demand is divided into six secondary indicators, and different tertiary indicators are divided under each secondary indicator. Through simulation analysis, it is confirmed that the improved algorithm proposed in this paper converges faster and finds the best path most. At the same time, the weight of the urban national sports fitness demand index is calculated.

## 1. Introduction

The ability to deal with public health emergencies is an urgent need to maintain national security and social stability. Timely and stable responses to public health emergencies are related to national security and development and the overall stability of the economy and society. If it is not handled properly and controlled effectively, not only the people's living standards and quality will be greatly affected but also people's panic will be caused, and the whole society will pay a heavy price. Improving the ability to deal with public health emergencies is the internal requirement to improve the national governance ability. Preventing and responding to public health emergencies is a complex and highly interrelated systematic project, which is a major test of the national governance system and governance ability.

With the improvement of the national economic level, the public's health awareness has also been significantly enhanced. At present, people are eager to improve their physical quality by participating in physical exercise. Therefore, the social demand for physical fitness is also accumulating [1]. Moreover, with the development of competitive sports, people began to pay attention to the development of sports and have a certain demand for sports products and venues. At present, in the research on sports fitness demand, the early research mostly emphasized the necessity and inevitability of health demand and also made it clear that sports health demand can bring a lot of economic value to the society [2]. In the relevant literature on demand content, in addition to analyzing the inevitability of sports health demand, the research on education also began to become a hot spot. With the acceleration of the aging process, the universal public health mode has been popularized [3]. Some scholars have also analyzed the differences in mass sports fitness needs and believe that there are great differences in the development of competitive sports between urban and rural areas, and the suburbs have great advantages in organizing events and activities. In these studies, qualitative analysis is mostly used, and quantitative questionnaire survey is mainly used, which is lack of predictability [4]. Based on this, this paper studies the prediction method of urban national health sports demand based on the ant colony algorithm.

This paper mainly studies and analyzes the urban national sports fitness demand prediction based on the ant colony algorithm, which is mainly divided into four chapters. Chapter 1 focuses on the research background and overall framework of this paper. The second part focuses on the research methods of demand forecasting at home and abroad and the application of the ant algorithm. The third chapter constructs the urban national sports fitness demand prediction, uses the fuzzy algorithm to layer the fitness demand prediction and calculate the weight, and improves the ant colony algorithm on the fuzzy analysis to realize the rapid calculation of the weight. The fourth chapter carries out simulation analysis, verifies the effectiveness of the algorithm proposed in this paper through the indicators such as convergence speed, convergence result, and error, and calculates the weight of the prediction index of urban national sports fitness demand.

Compared with the previous research results, the innovation of this paper lies in the analysis of research methods. Most of the previous studies used the literature method or questionnaire survey method, which is lack of accuracy and heavy workload. This paper proposes to use the ant colony algorithm to realize demand prediction analysis. Through the analysis of previous literature, the national sports fitness demand is divided into multiple secondary indicators, and the secondary indicators are divided into different tertiary indicators. Ant colony algorithm is used to improve the fuzzy algorithm and calculate the weight of tertiary indicators, which can compare and analyze the importance of different indicators. Then, it analyzes the concentrated performance of national fitness demand, which has a certain reference significance for improving the construction of stadiums and sports culture development.

## 2. Related Work

In recent years, there are many researches on demand forecasting, and some scientific research achievements have been made [5]. In the research and analysis, Alireza et al. used the ant colony algorithm to analyze the highway network of Kerman province, the largest province in Iran, which can identify the existing bottlenecks and predict the potential bottlenecks in the future [6]. Fan y et al. proposed a new model with unservice requirements by relaxing the requirements of meeting constraints, designed an algorithm based on distributed ant colony optimization (ACO), and made some specific modifications to it, using the average cost-saving percentage of each bicycle as a measure to evaluate the performance of our method in reducing costs [7]. Prasad et al. designed a method combining multistage multivariable empirical mode decomposition with ant colony optimization and random forest (i.e., MEMD-ACO-RF) to predict monthly solar radiation (RN). After calculating multivariable IMF, the ant colony optimization (ACO) algorithm was used to determine the best feature based on IMF for model development by combining the historical lag data at (*T*) − 1). The RF model is applied to the selected IMF to predict monthly RN [8]. In price reservation, Meng et al. proposed a parametric pricing method to formulate the pricing variables representing the pricing factors, calculated the pricing variables according to VMM and the regression relationship between the pricing variables and the price, and proposed a support vector regression (SVR)-integrated price prediction based on ant colony optimization algorithm (ACO) [9]. In climate research, Chaudhuri S et al. introduced swarm intelligence in the form of ant colony optimization (ACO) technology to calculate pheromone deposition on the path of the tropical cyclone and then used a neural network to predict the maximum sustained wind speed of cyclone over the Bay of Bengal (NiO) in the northern Indian Ocean [10]. In the research and analysis, Wan young et al. took baseball, bicycle, golf, and hiking club members as the research objects and analyzed the consumption tendency of sporting goods of activity participants from multiple dimensions [11]. In their research, Zhang *y* and others proposed a neural network sports load prediction model combined with the ant colony algorithm. The global search ability of the ant algorithm is used to determine the initial weight of the neural network, and the weight is further adjusted on the basis of neural network gradient descent to find the global best advantage. In the experiment, a three-layer BP neural network is used. It absorbs the advantages of the ant colony algorithm and neural network and has obvious advantages [12].

To sum up, it can be seen that there are many research methods related to demand forecasting, including cluster analysis, ant colony algorithm, and vector machine. In terms of research objects, in addition to theoretical research, demand forecasting research has a wide range of applications, such as logistics model, electricity, and transportation. However, there are few studies on sports, and there are few studies on the prediction of mass sports fitness demand. The prediction of sports demand is only involved and not in-depth. On the other hand, the existing prediction of physical exercise demand is generally based on a questionnaire survey, and the combination with an algorithm is generally related to site selection. Few studies can combine ant colony algorithms to construct sports health demand prediction.

## 3. Methodology

### 3.1. Neural Network Algorithm Based on Ant Colony Algorithm

The analytic hierarchy process is widely used in evaluation model, but this algorithm has a slow convergence speed and is easy to fall into a local minimum. This paper studies the use of the ant colony algorithm to improve the urban national sports fitness demand analysis. Ant algorithm simulates the ant's lost behavior and the ability to find the best nearest road, makes full use of the mechanism of selection, update, and coordination, and finds the optimal solution through the information exchange between individuals. Therefore, the ant colony algorithm is the algorithm that is most easy to find the better solution [13]. This paper uses the ability of the ant colony algorithm to add pheromone to each weight and uses the mean square error to simulate finding the optimal weight combination. Assuming that the number of ants is *m*, the obtained component is regarded as a vertex, and each vertex is a component. There are *ki* connecting lines between the *i* and *i*+1 vertices, which means that the value of the component is within this range [14]. Assuming that the pheromone on the *j* route at *t* time is *t*_*ij*_(*t*), the ant starts from this vertex, reaches the next vertex according to the strategy, and finally reaches the *n* vertex. The path that the ant passes through is a scheme. Assuming that the probability of ant transfer is expressed by *P*, the formula is

(1) $$\begin{array}{c} P_{ij}^{k}\left(t\right)=\left\{\frac{t_{ij}^{\alpha }\eta_{ij}^{\beta }\left(t\right)}{\sum_{0}r\in {\text{allowed}}_{k}t_{ij}^{\alpha }\eta_{ij}^{\beta }\left(t\right)},\;j\in {\text{allowed}}_{k}\right), \end{array}$$

where *η* belongs to heuristic information and represents visibility, *t* represents the strength of residual pheromone, and *P* represents the probability of ants choosing this path.

The path selected by the ant in the next step can be expressed as allowed_*k*_={*n* − tabu_*k*_}. After a period of time, a cycle is completed, and the pheromone of the path will change. The formula is adjusted to

(2) $$\begin{array}{c} t_{ij}\left(t+1\right)=\left(1-p\right)t_{ij}\left(t\right)+p\Delta t_{ij}\left(t,t+1\right),\\ \Delta t_{ij}\left(t,t+1\right)=\sum_{k=1}^{m}\Delta t_{ij}^{k},\;\left(t,t+1\right), \end{array}$$

where *p* represents the pheromone volatilization coefficient, which can reduce the continuous accumulation. The value range is 0∼1, and Δ*t* represents the pheromone left by the ant after selecting a path. In this formula, due to different algorithms, it is divided into three types, namely,

(3) $$\begin{array}{c} \Delta t_{ij}^{k}\left(t,t+1\right)=\left\{\begin{array}{c} Q,\text{ cycle passes through I and J},\\ 0,\text{else}, \end{array}\right.\\ \Delta t_{ij}^{k}\left(t,t+1\right)=\left\{\begin{array}{c} \frac{Q}{d_{ij}},\text{ cycle passes through I and J},\\ 0,\text{else}, \end{array}\right.\\ \Delta t_{ij}^{k}\left(t,t+1\right)=\left\{\begin{array}{c} \frac{Q}{L_{k}},\text{ cycle passes through I and J}.\\ 0,\text{else}. \end{array}\right. \end{array}$$

The first two algorithms release pheromones during construction, and the third one releases pheromones after completion [15]. The longest path traveled by ants is used as the overall information, and the pheromone strength is constant, which will affect the convergence speed.

When the ant colony algorithm is used for demand forecasting, it is mainly used to complete the premise work to optimize the weights and thresholds of the neural network, narrow the range, and then accelerate the convergence in combination with the improvement of the neural network [16], as shown in Figure 1. Before the implementation of the ant colony algorithm, each weight variable of the neural network is segmented. The ant passes through each weight vector, selects a value in the definition domain, completes the selection of weight variables, constructs a group of weights, inputs the sample data, and updates the pheromone after calculating the error. Using the ant algorithm can improve performance and deal with a wide range of data sets [17]. In order to better deal with the data, we need to deal with the prior knowledge of the problem. In order to better explore the path, the principle of random proportion is adopted. The global update is carried out on the optimal ant path. After each cycle, only the path traveled by the ant is enhanced. In this way, under the volatilization mechanism, other paths are continuously reduced, the difference between the optimal path and other paths is completed, the optimal path is reached more quickly, and the efficiency of the algorithm is quickly improved [18]. Specifically, when selecting the path, the random proportion principle is used, and the ants at the node use the rules to select the point. The formula is

(4) $$\begin{array}{c} s=\left\{\begin{array}{c} \arg\underset{u\in {\text{allowed}}_{k}}{\max}\left\{{\left[t\left(i,u\right)\right]}^{a}\left[\eta \left(i,u\right)\right]\beta \right\},q\leq q_{0},\\ s,\text{else,} \end{array}\right) \end{array}$$

where *i* represents the node, *q* represents the randomly generated value, ranging from 0 to 1, and *S* represents the proportion rule. This random rule can use the prior knowledge about the problem to limit the search to the range of the optimal solution and can use the proportional rule to know the relative importance. When ants choose the path, they give priority to the path with the shortest path and the most pheromones. It is assumed that the preset parameters are expressed by *a* and *b* to describe the relationship between heuristic information and pheromone concentration. After each cycle is completed, the optimal information degree is enhanced, and the global optimal path forms a weight sequence [19]. The minimum error of the sequence is calculated. Assuming that the volatilization parameter is expressed by *P*, the pheromone update formula can be expressed as

(5) $$\begin{array}{c} t\left(i,s\right)=\left(1-p\right)t\left(i,s\right)+p\Delta t\left(i,s\right),\\ \Delta t\left(i,s\right)=\left\{\begin{array}{c} \frac{Q}{E},\text{path belongs to the optimal path},\\ 0,\text{else}, \end{array}\right) \end{array}$$

where, if (*i*, *s*) belongs to the global optimal path, Δ*t*(*i*, *s*)=*Q*/*E*; otherwise, Δ*t*(*i*, *s*)=0.

In the application of a neural network based on the ant colony algorithm, the weights are initialized and divided first. According to the random ratio rules, the ants transfer and mark the passing points. When the ownership value is taken, a cycle is completed, and the recorded points form a group of weights to obtain the data and error. The pheromone is updated according to the global update strategy until the maximum evolution algebra is satisfied, and the adaptive learning rate improvement algorithm is used for further calculation. Through these calculations, the convergence speed of the algorithm can be quickly improved. However, due to the characteristics of the ant colony algorithm itself, the search speed is still slow, so it needs to be further improved to avoid premature [20]. After each cycle, only one ant pheromone is set to update to find the optimal solution for the current cycle. In order to avoid stagnation, all elements are limited to a fixed interval. Pheromone trajectory rules can be expressed as

(6) $$\begin{array}{c} t_{ij}\left(t+1\right)=\rho t_{ij}\left(t\right)+\Delta t^{{\text{best}}_{ij}}, \end{array}$$

where *t*_max_ represents the trajectory and *f* represents the iterative optimal solution. The pheromone evaluation mechanism is further updated, and the formula is expressed as

(7) $$\begin{array}{c} t_{ij}^{*}\left(t\right)=t_{ij}\left(t\right)+\delta \left(t_{\max}\left(t\right)-t_{ij}\left(t\right)\right), \end{array}$$

where *δ* represents the retention of previous pheromones, ranging from 0 to 1. When *δ*=1, it indicates trajectory initialization, and when *δ*=0, it indicates a complete shutdown mechanism. Under this mechanism, the pheromone distribution at stagnation can be obtained.

In the incremental allocation of information, different paths get the same enhancement, and the search results are different in different sections. For better paths, larger pheromones need to be allocated, and for worse paths, smaller pheromones need to be allocated. Assuming that the total number of occurrences of the path in the search cycle is *k*, there is

(8) $$\begin{array}{c} \Delta t_{ij}=\frac{\sqrt[{5}]{k}}{f\left(s^{\text{best}}\right)}, \end{array}$$

where *f*(*s*^best^) represents the optimal path length. In order to speed up the process and promote ants to gather in the optimal path as soon as possible, weakening the worst solution is considered. On the nonoptimal and worst paths, the pheromone is adjusted according to the following formula:

(9) $$\begin{array}{c} t_{ij}\left(t+1\right)=\rho t_{ij}\left(t\right)-\Delta t^{{\text{worst}}_{ij}}, \end{array}$$

where *ρ* is the parameter, and the value is 0.5.

### 3.2. Fitness Demand Prediction Model

In the new era, the evaluation index system of urban national sports fitness needs to meet the requirements of scientificity, operability, and reliability. The corresponding index values of many indicators need to be able to be analyzed quantitatively. In the demand for sports health, it is necessary to put forward some data that are easy to obtain but cannot obtain specific indicators and reasonably match some indicators. In the evaluation of national sports fitness needs, we hope to cover most cities. However, due to the great differences in economic levels, many indicators should take the average value. In the selection of indicators, we should combine the professionalism and practicality of sports and improve adaptability at the same time.

Combined with the construction of physical fitness, the construction level of physical fitness is the objective subject, and there are six secondary indicators, namely fitness demand, entertainment demand, talent demand, product demand, social demand, and venue demand. Each indicator corresponds to the tertiary indicators, as shown in Figure 2. Fitness needs include exercise times and practice, need for venues, and need for environment and clubs. Entertainment needs are divided into the hope that projects will be valued, need more practice, need to improve their level, watch sports projects, and participate in sports teams. Talent needs are divided into high-level athletes' joint participation, sports instructors, managers, sports talents, and sports coaches. The demand for sports products is divided into purchasing sports products, increasing product consumption, better shopping, and liking sports clothes. The social demand is divided into enhancing the feelings with friends through sports, learning to communicate, increasing the scope of making friends, and requiring the joint participation of friends. The venue demand is divided into more sports places, reducing unnecessary places, open places, more sound surrounding settings, and more space for movement.

Fuzzy comprehensive evaluation method is an improvement of the previous mandatory evaluation. This method divides the evaluation area into different types and makes weighted analysis on each index, which belongs to the evaluation method of the combination of qualitative analysis and quantitative analysis. The fuzzy evaluation method is more effective for complex systems. When applied, the definition model is inputted, the weight coefficient of each index by the analytic hierarchy process is calculated, and the weight of each index is expressed by *w*_*i*_. The weight of secondary indicators is represented by *w*_*ij*_, and the weight of three-pole indicators is represented by *w*_*ijk*_. The indexes of sports demand are dimensionless to ensure that different indexes can be compared, and the index analysis model is obtained. All indicators are positive, so the fuzzy membership function is used to standardize each indicator. The function is

(10) $$\begin{array}{c} \Phi \left(e_{ij}\right)=\left\{\begin{array}{c} 1,e_{ij}=M_{j},\\ \frac{e_{ij}-M_{j}}{M_{j}-m_{j}},\;m_{j}<e_{ij}<M_{j},\\ 0,e_{ij}=m_{j}, \end{array}\right) \end{array}$$

where *e*_*ij*_ represents the specific attribute value of the regional indicator, *M*_*j*_ represents the maximum value of the indicator, and *m*_*j*_ represents the minimum value of the indicator. This quantitative method can ensure the comparability between different indicators. The larger the value, the closer the actual value is to the maximum value. The difference between 1 and 1 is the difference in the maximum demand. The following formula is used to calculate the sports hypothesis:

(11) $$\begin{array}{c} Y=f\left(i\right)=\sum_{j=1}^{48}\Phi \left(e_{ij}\right)w_{j}, \end{array}$$

where Φ represents the fuzzy membership function value of the index.

## 4. Result Analysis and Discussion

### 4.1. Simulation Analysis of Ant Colony Algorithm

TSPLIB data are selected, the experimental parameter *α* is 1, *β* is 3, *ρ* is 0.95, *C* is 0.01, *P*_*best*_ is 0.05, and the number of iterations is 3000 test 10 times each time and calculates the average value. The calculation results are shown in Figure 3. It can be seen from the data in the figure that the error between the algorithm proposed in this paper and the optimal solution is the smallest in different examples, and the number of times to find the optimal solution is also the largest.

The optimal solution data published by TSPLIB are analyzed, and the optimal solution data are found by the algorithm in this paper and calculated the error, as shown in Figure 4. It can be seen from the figure that the error is less than 1%, which proves the effectiveness of the algorithm.

The robustness of the algorithm is analyzed in MATLAB 7. When the training error result reaches 0.1, it is considered that the training is correct; otherwise, the training is continued. The weight variables are changed and modified in order to get better results. This paper tests the algorithm and iterates the loop. The convergence images are compared and analyzed, the error and convergence time are analyzed, and the internal initial weight is improved. The comparison results of internal improved convergence are shown in Figure 5. It can be seen from the data in the figure that the algorithm proposed in this paper can greatly improve the convergence.

The learning rate is set as 0.9 and 0.0001 as too small values and analyzes the correction results of the convergence effect, as shown in Figure 6. From the changes in the figure, it can be seen that the algorithm proposed in this paper has an obvious convergence effect.

The analysis of the convergence time and results of the algorithm is shown in Figure 7. From the data in the figure, it can be seen that the convergence speed of the algorithm proposed in this paper is significantly improved. The scenic spot algorithm needs 1000 iterations to achieve the required accuracy. The improved algorithm can save 2/3 of the time and have less error.

### 4.2. Forecast and Analysis of Fitness Demand

The prediction indexes of urban national fitness demand are screened and revised, the optimal weight combination is studied and found, an adaptive algorithm is learned to avoid premature convergence, the performance of the ant colony algorithm is improved, and the national fitness demand is predicted and analyzed, which is divided into two-level indexes and three-level indexes. By comparing the indicators, a judgment matrix is built, the weight calculation is completed, and the final weight calculation result is obtained. In the process of index data processing, because the index itself has qualitative and quantitative analysis, it is necessary to process the data. All original indicators are quantified to ensure comparability between different indicators. The weight calculation is completed by MATLAB software, and the weight coefficient of each index is obtained through a consistency test.

Among the secondary indicators, the weight coefficient of fitness demand is 0.1, entertainment demand is 0.1, talent demand is 0.2, product demand is 0.3, social demand is 0.1, and venue demand is 0.2. Each indicator corresponds to three-level indicators. Under the demand of fitness, the exercise weight coefficient of the three-level indicators is 0.3. The required site weight coefficient is 0.3, the required environment weight coefficient is 0.3, and the club weight coefficient is 0.1. Under the secondary indicators of entertainment demand, the tertiary indicators hope that the project will be paid attention to. Under the talent demand index, the weight coefficient of high-level athletes participating in the three-level index is 0.2, the weight coefficient of sports instructors is 0.2, the weight coefficient of managers is 0.3, the weight coefficient of sports talents is 0.2, and the weight coefficient of sports coaches is 0.1. Under the secondary index of sports products, the weight coefficient of the tertiary index for purchasing sports products is 0.2, the weight coefficient of increased product consumption is 0.2, the weight coefficient of better stores is 0.2, and the weight coefficient of favorite sports clothing stores is 0.4. Under the social needs of the secondary indicators, the weight coefficient of the tertiary indicators is 0.3, the weight coefficient of learning to communicate is 0.2, the weight coefficient of increasing the range of making friends is 0.2, and the weight coefficient of requiring the joint participation of friends is 0.3. Under the site demand of secondary indicators, the weight coefficient of more stadiums in tertiary indicators is 0.3, the weight coefficient of reducing unnecessary places is 0.1, the weight coefficient of open places is 0.2, the weight coefficient of surrounding settings is 0.3, and the weight coefficient of larger sports space is 0.1.

## 5. Conclusion

This paper studies the demand prediction of urban national sports fitness based on the ant colony algorithm and puts forward the shortcomings of the fuzzy analytic hierarchy process. The research adopts an ant colony algorithm to improve, increases pheromone for each group of weight, updates information with mean square error, and finds the optimal weight combination. And learn from the adaptive algorithm to avoid premature convergence, improve the performance of the ant colony algorithm, predict and analyze the demand for national fitness sports, and divide it into two-level indicators and three-level indicators. Through analysis, it is proved that the algorithm proposed in this paper has good convergence, effectiveness, and error performance, and the superiority of the algorithm is proved. It should be pointed out that there are many demand forecasting algorithms. This paper focuses on the analysis of the ant colony algorithm. At present, there is little research on the application of the algorithm in sports demand, which needs to be improved in combination with the specific problems in parameter selection. However, in the simulation analysis of this paper, the test is carried out in an ideal state. Affected by economic and environmental conditions, many data may not be continuous and complete. Therefore, the analysis of the algorithm needs to be further strengthened in future research.

## Figures and Tables

**Figure 1:** Network optimization flow chart of ant colony algorithm.

**Figure 2:** Sports fitness demand index system.

**Figure 3:** Performance comparisons of 4 algorithms.

**Figure 4:** Error analysis.

**Figure 5:** Convergence analysis of the algorithm.

**Figure 6:** Correction result of excessive learning rate.

**Figure 7:** Convergence time and results of the algorithm.

## Data Availability

The data used to support the findings of this study are available from the corresponding author upon request.
